# Research on Haze Image Enhancement based on Dark Channel Prior Algorithm in Machine Vision

This article has been retracted.

**DOI:** 10.1155/2022/3887426

**Published:** 2022-07-07

**Authors:** Dan Li, Jinping Sun, Hongdong Wang, Hanqin Shi, Weiwei Liu, Likai Wang

**Affiliations:** ^1^School of Information Engineering (School of Big Data), Xuzhou University of Technology, Xuzhou, Jiangsu, China; ^2^Traffic Police Detachment of Xuzhou Public Security Bureau, Xuzhou, Jiangsu, China

## Abstract

According to the characteristics of foggy images, such as high noise, low resolution, and uneven illumination, an improved foggy image enhancement method based on dark channel priority is proposed. First, the new algorithm refines the transmittance and optimizes the atmospheric light value and converts the restored image to HSV space. Second, the brightness *V* component is enhanced by MSRCR algorithm improved by bilateral filtering, and the saturation S is improved by adaptive stretching algorithm. Finally, the image is converted from HSV space to RGB space to complete image enhancement. The new method solves the problems of that the color of large area is uneven and the overall color of the image is dark when the traditional dark channel prior method is used to remove fog. The experimental results show that from subjective evaluation and quantitative analysis the new algorithm overcomes the shortcomings of noise amplification and edge blur when the conventional enhancement algorithm enhances the image. It can improve image darkening and avoid image distortion in JPEG, BMP, GIF, PNG, PSD, and TIFF formats. By comparing with other image enhancement algorithms, the improved algorithm performs better than DCP, SSR, MSR, MSRCR, and CLAHE algorithm in PSNR, SSIM, and IE evaluation indexes. It has a good effect on preserving the edge information and has good adaptability and stability for heavily polluted haze image enhancement.

## 1. Introduction

With the gradual aggravation of environmental pollution, more and more cities frequently appear haze. Due to the low contrast and saturation of the image collected in foggy days, the color is prone to offset and distortion, which has a bad impact on the computer vision system relying on image information. Therefore, how to improve the image quality through a simple and effective image defogging method is a hot topic.

The commonly used image defogging methods mainly include image enhancement and image restoration. However, the former does not consider the image degradation caused by fog, and directly uses some image enhancement algorithm to remove fog. It is mainly divided into global image enhancement and local image enhancement. Global image enhancement methods include global histogram equalization algorithm, wavelet, and multiscale analysis method, Retinex algorithm based on color constancy principle. Local image enhancement methods include local histogram equalization algorithm, local contrast enhancement algorithm, and local variance enhancement algorithm. Image enhancement realizes defogging by high-lighting the details of the image, ignoring the essence. Based on the physical model of atmosphere, the image restoration method can get the parameters by applying prior conditions to remove fog. The model is used to estimate the model parameters and then restore the image. The restoration of fog image based on physical model mainly includes partial differential equation based, depth relationship based and prior information. In recent years, some experts have put forward more and more defogging methods based on the above ideas, and have made some achievements.

In order to solve the problem of blocking effect in the restored image of large uniform regions such as sky, Tufail et al. [1] proposed a single image defogging technique based on dark channel to estimate the atmospheric light, and reconstruct the fog free image using atmospheric light and transmission image. According to the density of fog, the transmission image is adaptively selected to reconstruct the image, and the transmission image is refined by the combination of Laplacian filter and pilot filter. Salazar-Colores et al. [2] proposed a image restoration algorithm based on morphological reconstruction to solve the problem of haze, smoke and fog caused by suspended particles (such as dust, carbon, and water droplets) in the air which will lead to image degradation. The experimental results were evaluated qualitatively. Chen et al. [3] proposed an improved blind image deblurring algorithm and solved the ringing effect caused by incorrect fuzzy kernel estimation. High-pass filter improved the image quality. The method of combining super Laplacian priori and dark channel priori is used to estimate the potential clear image. The accurate blur kernel is estimated by alternating iteration from coarse to fine. A deconvolution method based on Laplacian prior and regularization prior is used to restore the clear image. Raikwar and Tapaswi [4] proposed that the accuracy and effectiveness of single image deblurring depends on the accuracy of transmitted light and atmospheric light. The problem of transmission estimation is transformed into the estimation of minimum color channel difference between blurred image and nonblurred image, and a nonlinear model is proposed to estimate the bound function, so as to realize the accurate estimation of transmission. Anan et al. [5] proposed a framework based on the segmentation of sky and nonsky regions to restore the sky and nonsky parts, respectively. The sky part is restored by contrast limited adaptive histogram equalization (CLAHE) method, and the nonsky part is restored by improved DCP method and fused to get the final image. Wang et al. [6] proposed an image-defogging algorithm based on different color wavelength compensation. It can restore the haze free image and reduce the color distortion of the bright area. Zou et al. [7] proposed a new defogging algorithm for blurred images. First, the logarithmic pilot filter was used to estimate the ambient light, which retained the characteristics of the image in the bright light source region and improved the fuzzi-ness of the dark light source region. Second, aiming at the disadvantage that the brightness of dark channel prior and bright channel prior is too high, the multichannel prior method is introduced. Finally, an adaptive transmission value calculation method based on multiple priors is proposed.

In recent years, image-defogging algorithm based on neural network has made rapid development. Li et al. [8] combined transmittance and atmospheric light into one variable and proposed a multiscale network structure (AOD-et). The network results eliminate the error of separate training of atmospheric light and transmittance and achieve better restoration effect. But the result of the algorithm is dark. Liu et al. [9] proposed a residual network structure, combined with the foggy image and its hypothesis or prior information, to estimate the transmittance, and then get the restoration results. However, this method takes the composite image as the training set, so the stability of the restoration effect is poor, and the applicability for real outdoor foggy images is low. Chen et al. [10] proposes a hybrid-learning algorithm DehazeNet based on patch graph, which combines the two strategies by using a hybrid learning technology including patch graph and dual attention generation antagonism network. Sharma et al. [11] studies the main problems of the image processing technology based on physical model, decomposes the existing deep learning methods into three categories: convolution neural network, recurrent neural network and generation confrontation network, and compares their advantages and disadvantages. However, it does not consider the nature of image degradation, resulting in the trained model is full of uncertainty for fog image restoration in real environment.

Therefore, based on the single image dark channel prior defogging algorithm, this paper analyzes the degradation process of foggy image, and improves the method based on dark channel prior algorithm according to the image haze distribution characteristics. In view of the uneven thickness of cloud and fog in the original image, a linear attenuation model based on the fog concentration distribution is established to modify the atmospheric light value and transmittance. By refining the atmospheric transmittance, the atmospheric light value estimation is optimized to improve the clarity of the output image. In view of the situation that the brightness of the restored image is reduced, the image is transferred to HSV space, the *S* component is stretched linearly, and the brightness *V* component is processed by MSRCR algorithm. The restored image is enhanced twice. Finally, the image is transformed back to RGB space to realize the defogging enhancement.

## 2. A Priori Method of Dark Channel

### 2.1. Atmospheric Scattering Model

When the light meets the suspended particles in the atmosphere, part of the incident light will be scattered by the particles, so that the light intensity will be weakened [12–14]. Therefore, each suspended particle in the gas can be regarded as a separate scatterer. Generally speaking, the scattering intensity does not affect each other [15, 16]. According to the study of atmospheric scattering mechanism, Mie scattering mechanism can be used to analyze the scattering effect of dust, mist, fog, dense fog, and other adverse weather conditions [17, 18]. The atmospheric scattering model is expressed as follows:

(1) $$\begin{array}{c} I\left(x\right)=J\left(x\right)t\left(x\right)+A\left(1-t\left(x\right)\right). \end{array}$$

In the above formula, *x* is the position coordinate of the current pixel, *I*(*x*) is the illumination intensity at *x* obtained at the observation point, *t*(*x*) is the transmittance from *x* to the observation point, which reflects the ability of light to penetrate the medium. *A* is the global atmospheric light value, and *J*(*x*) is the intensity of the reflected incident light of the target in the detection scene. *A*(1 − *t*(*x*)) is the atmospheric light component, that is, the light intensity of ambient light scattered by haze and other media to the observation point. *J*(*x*)*t*(*x*) is called direct attenuation, indicating the attenuation degree of reflected light at *x* in the atmosphere. The above formula can also be written as follows:

(2) $$\begin{array}{c} J\left(x\right)=\frac{I\left(x\right)-A\left(1-t\left(x\right)\right)}{t\left(x\right)}. \end{array}$$

The key to solve the problem of clear and fog free image *J*(*x*) is how to estimate the global atmospheric light value *A* and transmittance *t*(*x*). *t*(*x*) can be expressed as follows:

(3) $$\begin{array}{c} t\left(x\right)=e^{-\beta d\left(x\right)}. \end{array}$$

The above formula indicates that the contrast of the scene decreases exponentially with the increase of the depth of field, *β* represents the scattering coefficient caused by light scattering and absorption by atmospheric particles. It is considered to be constant. *d* is the depth of field of the image.

### 2.2. Dark Channel Prior Theory

Image enhancement algorithm only takes into account the numerical level of operation [19–22], although it improves the image tone and contrast to a certain extent, but it does not go deep into the essence of defogging, so it is not enough to only use image enhancement algorithm, image enhancement based on image restoration can achieve good results [23–25]. Based on the physical model, the dark channel prior theory deduces the unknown parameters of the model with reasonable assumptions to re-store the fog free image.

In the dark channel prior method, when the foreground part of the sky region is removed from the image, there will always be a certain color channel of at least one pixel with a very low intensity value, which is called dark primary color. For any input image, the dark primary color points can be solved by formula:

(4) $$\begin{array}{c} J^{\text{dark}}\left(x\right)=\underset{c\in \left\{r,g,b\right\}}{\min}\left(\underset{y\in \Omega \left(x\right)}{\min}\left(J^{c}\left(y\right)\right)\right). \end{array}$$

Among formula (4) *J*^dark^(*x*) represents the dark channel image of the image, and for the fog free image of the nonsky region, the dark channel of *J*^dark^(*x*) tends to 0, Ω(*x*) represents a square sliding window centered on pixel *x*, and *J*^*c*^*r*efers to one of several channels of color image. In the haze image, because the particles make the atmosphere scatter, the brightness of the image is increased, and the contrast is decreased, so that the corresponding dark channel value no longer tends to 0. For haze image processing, it is assumed that the atmospheric light value *A* is given. Suppose a window centered on pixels *x*, the transmissivity in Ω(x) is constant, denoted as $\tilde{t}\left(x\right)$. The physical model of fog map is simulated, and the size of local area is set as Ω(*x*). As shown in formula.

(5) $$\begin{array}{c} \underset{y\in \Omega \left(x\right)}{\min}\left(I^{c}\left(x\right)\right)=\tilde{t}\left(x\right)\underset{y\in \Omega \left(x\right)}{\min}\left(J^{c}\left(x\right)+A^{c}\left(1-\tilde{t}\left(x\right)\right)\right). \end{array}$$

The atmospheric light value *A* is not 0, and divide both sides of formula (5) by *A*^*c*^, the minimum value filtering is made on three channels.

(6) $$\begin{array}{c} \underset{c}{\min}\left(\underset{y\in \Omega \left(x\right)}{\min}\left(\frac{I^{c}\left(x\right)}{A^{c}}\right)\right)=\tilde{t}\left(x\right)\underset{c}{\min}\left(\underset{y\in \Omega \left(x\right)}{\min}\left(\frac{J^{c}\left(x\right)}{A^{c}}\right)\right)+\left(1-\tilde{t}\left(x\right)\right). \end{array}$$

According to the prior principle of dark channel, the dark primary color value of clear fog free image *J*^*c*^(*x*) tends to 0, and the transmittance $\tilde{t}\left(x\right)$ is as follows:

(7) $$\begin{array}{c} \tilde{t}\left(x\right)=1-\underset{c}{\min}\left(\underset{y\in \Omega \left(x\right)}{\min}\left(\frac{I^{c}\left(x\right)}{A^{c}}\right)\right). \end{array}$$

So far, the estimated value of transmittance *t*(*x*) is generally correct, but directly used for image defogging will produce halo in some cases. We can use the filter to estimate more precise transmittance, filter out halo, and obtain better defogging effect. Because there are some particles in the clear sky in real life, we can still feel the fog when watching distant objects, so we can keep a certain degree of fog when removing the fog. A constant *ω*(0 < *ω* ≦ 1) is introduced into formula (8), set up *ω* = 85.

(8) $$\begin{array}{c} \tilde{t}\left(x\right)=1-\omega \underset{y\in \Omega \left(x\right)}{\min}\left(\underset{c\in \left\{r,g,b\right\}}{\min}\frac{I^{c}\left(y\right)}{A^{c}}\right)\left(\omega \in \left(0,1\right]\right). \end{array}$$

In the dark primary color image of haze image, the lower the transmittance is, the thicker the fog is and the brighter the image is. That is to say, when the transmittance tends to 0, the brightness value of the point with the densest fog is the atmospheric light value. Therefore, the first 0.1% of the highest brightness value in the dark channel image is selected as the point with the highest fog. In the original fog map, the highest value of each channel corresponding to these points is selected as the atmospheric light value *A*. Combined with the estimated transmittance $\tilde{t}\left(x\right)$ and atmospheric light value *A*, the restored fog free image is obtained.

(9) $$\begin{array}{c} J\left(x\right)=\frac{I\left(x\right)-A}{\tilde{t}\left(x\right)}+A. \end{array}$$

Although the defogging method based on the principle of dark primary color can restore fog free image more realistically, it has some limitations. When processing the image with sky area or high brightness area, the depth of field is wide, the light of vehicle, large sky area and white object will affect the estimation of atmospheric light value *A*, resulting in poor defogging effect and color block effect in the sky area. The results show that the defogging image has obvious white edge effect, which is caused by the rough transmittance. In addition, the defogging images are generally dark. Aiming at the color block effect of dark channel defogging, this paper solves it by reasonably estimating the transmittance and atmospheric light value, and solves the problem of dark tone by MSRCR algorithm enhancement.

## 3. New Image Defogging Algorithm

In view of the above problems in fog image enhancement, this paper calculates the dark primary color image based on the dark channel principle [26–29], optimizes the calculation process of transmittance *t*(*x*) and the estimation of atmospheric light value *A*, and then restores the image to HSV space. In RGB color space, the relationship between the values of the three-color components and the generated colors is not intuitive. In HSV color space, it is easier to track objects of a certain color than RGB. It is often used to segment objects of a specified color. The *V* component is enhanced by MSRCR algorithm, and the *S* component is linearly stretched, which can improve the image clarity and effectively alleviate the phenomenon of object edge blur and halo, avoid image darkening, maintain the original color of the image, and enhance the brightness and contrast details of the image. The algorithm flow is shown in Figure 1 below.

### 3.1. Improvement of Atmospheric Light Value

In the above inference, the atmospheric light *A* should be estimated before the transmission rate $\tilde{t}\left(x\right)$ estimation, and its estimation accuracy greatly affects the final image restoration. He and Sun [30] extracted the first 0.1% pixels in the dark channel according to the brightness size, and then took the maximum value of the original image corresponding to the pixel as the value of *A*. However, this method may make the *A* value of each channel close to the maximum pixel value 255, resulting in the color deviation, the brightness distortion or a large number of color spots in the processed image. In order to better estimate the value of atmospheric light *A*, this paper proposes an optimization method of atmospheric light based on the fog concentration distribution.

First, the sky and nonsky regions are segmented by OTSU image segmentation method [31–34], and the average intensity value of the sky region of the original image after segmentation is taken as the estimated value of *A*. Since the depth of field of the sky region can be regarded as infinite, that is *d*(*x*)⟶+*∞*, we can know *t*(*x*) ≈ 0, taking it into equation (3), It can be seen that:

(10) $$\begin{array}{c} I\left(x\right)\approx A. \end{array}$$

In the above formula, *A* is the brightness value of the maximum fog area, so it is reasonable to take the average intensity of the sky area as the value of atmospheric light *A*. That is,

(11) $$\begin{array}{c} A^{c}=\underset{c\in \left\{r,g,b\right\}}{\text{mean}}I_{s}^{c}\left(y\right), \end{array}$$

Where *I*_*s*_^*c*^ represents a color channel in the sky, and mean_*c*∈{*r*, *g*, *b*}_ is the average filter, the final transmissivity is obtained by introducing the above equation (8):

(12) $$\begin{array}{c} \tilde{t}\left(x\right)=1-\omega \underset{y\in \Omega \left(x\right)}{\min}\left(\min\frac{I^{c}\left(y\right)}{{\text{mean}}_{c\in \left\{r,g,b\right\}}I_{s}^{c}\left(y\right)}\right). \end{array}$$

### 3.2. Transmittance Estimation Based on Fog Concentration

In the process of atmospheric imaging, atmospheric light *A* foggy image *I*(*x*) and clear image *J*(*x*) are coplanar, and the mode length decreases in turn. Obtaining *J*_min_^*c*^(*x*) is the key to estimate the transmission. There is a certain attenuation relationship between foggy image and clear image. Wang et al. [35] proposed a linear attenuation model based on minimum channel, as shown in equation.

(13) $$\begin{array}{c} J_{\min}^{c}\left(x\right)=\frac{I_{\min}^{c}\left(x\right)-\text{Min}}{\text{Max}-\text{Min}}I_{\min}^{c}\left(x\right), \end{array}$$

Where Max is the maximum of *I*_min_^*c*^(*x*) and Min is the minimum of *I*_min_^*c*^(*x*). Under the condition of uniform distribution of fog concentration, this attenuation can reflect the relationship between the minimum channel of foggy image and clear image, but under natural conditions, the fog concentration of foggy image changes with the depth of field, so the above attenuation cannot accurately reflect the mapping relationship between the minimum channel.

It is found that, the fog concentration increases with the increase of depth of field. It can be considered that for a clear image, when affected by fog, the influence is different in the close range and depth of field. For the depth of field region, the degradation is more serious due to the influence of dense fog, that is, in the dense fog region, the attenuation from foggy image to clear image is more severe. Inspired by the linear attenuation model, a linear attenuation model based on fog concentration distribution is proposed in this paper. The expression is as follows:

(14) $$\begin{array}{c} J_{\min}^{c}\left(x\right)=\left[\gamma +W\prime \left(x\right)\right]\times I_{\min}^{c}\left(x\right), \end{array}$$

Where *γ* is the attenuation constant and *W*′(*x*)*W*′(*x*) is the adaptive fog concentration attenuation function. In order to accurately reflect the different attenuation speed in different fog concentration regions, the adaptive fog concentration attenuation function is defined as follows:

(15) $$\begin{array}{c} W\prime \left(x\right)=\frac{W_{\max}\left(x\right)-W_{\min}\left(x\right)}{2}. \end{array}$$

It can be seen from equation (15), in the region with high-fog concentration, *W*′(*x*) has a larger value, which makes *J*_min_^*c*^(*x*) have a stronger pixel value in the dense fog region. In the close range area, if *W*′(*x*)*W*′(*x*) is small, the intensity of *J*_min_^*c*^(*x*) is low, even close to 0. This is in line with the theory that dark channels tend to zero proposed by He and Sun [30]. In order to further reflect the attenuation difference between the dense fog and the close range area, the attenuation constant is introduced to compensate for the attenuation. In this paper, the value is the gray mean value of the fog concentration, that is:

(16) $$\begin{array}{c} \gamma =\text{mean}\left(W\left(x\right)\right). \end{array}$$

In conclusion, the transmittance can be expressed as follows:

(17) $$\begin{array}{c} t\left(x\right)=\frac{A-I_{\min}^{c}\left(x\right)}{A-\left[\gamma +W\prime \left(x\right)\right]\times I_{\min}^{c}\left(x\right)}. \end{array}$$

In order to eliminate texture, the transmission rate can be smoothed by bilateral filtering, and then the transmittance is obtained.

### 3.3. Combining Retinex Algorithm

The image after dark primary color processing is generally dark in visual effect, which can be improved by fusing Retinex algorithm [36, 37] after restoration. However, in practical application, Retinex algorithm is easy to produce halo at the edge when processing the edge part with large brightness difference in order to take into account the change of light in the image [38, 39]. When it enhances RGB model, it will ignore the relationship of three channels and may appear distortion. Therefore, the original restored image is transformed from RGB model to HSV model, and MSRCR image is enhanced and *S* component is stretched in HSV color space.

Retinex theory holds that the image formed in human eyes is formed by the object reflecting the light [40]. The color of the object itself has nothing to do with the external factors. What actually plays a role is the reflection ability of the object to various types of light sources. Therefore, the model consists of two parts, one is illumination component, the other is reflection component. The model expression of Retinex theory is as follows:

(18) $$\begin{array}{c} I\left(x,y\right)=R\left(x,y\right)\times L\left(x,y\right). \end{array}$$

*I*(*x*, *y*) is the final received image information; *R*(*x*, *y*) is the reflection component of the object, which usually has a lot of high-frequency information. It represents the reflection ability of the object itself to light, and has nothing to do with the light itself; *L*(*x*, *y*) is the illuminance component of light, usually a low frequency signal. It can be seen that the information of the object itself can be obtained by removing the illumination component from the final received image, so that the effect of image enhancement can be achieved. Based on this, the SSR algorithm [41, 42] transforms equation (18) into logarithmic domain, which is expressed as follows. Where *I*_*i*_(*x*, *y*) is the *i*-th color component of the input image, *R*_*i*_(*x*, *y*) is the output of the *i*-th color component, and the illumination component is convoluted with the image obtained by *F*(*x*, *y*):

(19) $$\begin{array}{c} R_{i}\left(x,y\right)=\log\;I_{i}\left(x,y\right)-\log\left[F\left(x,y\right)*I_{i}\left(x,y\right)\right]. \end{array}$$

The expression of Gaussian function is as follows:

(20) $$\begin{array}{c} F\left(x,y\right)=Ke^{-\left(x^{2}+y^{2}\right)/\sigma^{2}}. \end{array}$$

*σ* is the scale parameter used to adjust the dynamic compression range and color balance. *K* is the normalized constant and satisfies the equation ∬*F*(*x*, *y*)d*x*d*y*=1.

Since SSR cannot satisfy both dynamic range compression and color fidelity, a multiscale Retinex (MSR) [43, 44] is proposed, whose expression is

(21) $$\begin{array}{c} R_{i}\left(x,y\right)=\sum_{n=1}^{N}W_{n}\left\{\log\left[I_{i}\left(x,y\right)\right]-\log\left[I_{i}\left(x,y\right)*F_{n}\left(x,y\right)\right]\right\}, \end{array}$$

Where *W*_*n*_ is the weight factor of the nth scale, and satisfies ∑_*n*=1_^*N*^*W*_*n*_=1 and *N* represents the number of scales. By adjusting the weight factor and scale parameters, dynamic compression and tone reproduction can be achieved. The fog image enhancement algorithm based on MSR not only makes the details of the image clearer, the color fidelity higher, and the global contrast higher but also removes the large-scale convolution operation, suppresses the halo effect of the image, improves the operation efficiency of the algorithm, and can avoid the problem of uneven image enhancement of the traditional algorithm. Because the processing results will have color distortion, this paper introduces the MSRCR method [45, 46] of color recovery factor, and introduces the color recovery factor *C* on the basis of MSR. MSRCR algorithm has good color reproducibility, brightness constancy, and dynamic range compression. It has better image enhancement effect and more realistic color than MSR. The local contrast of the image processed by MSRCR algorithm is improved, and its brightness is similar to the real scene, so the image is more realistic under visual perception. The expression is as follows:

(22) $$\begin{array}{c} {\text{RMSRCR}}_{i}=C_{i}\left(x,y\right){\text{RMSR}}_{i}\left(x,y\right),\\ C_{i}\left(x,y\right)=\frac{\beta \left\{\ln\left(\alpha I_{i}\left(x,y\right)\right)\right.}{\sum_{n=1}^{N}I_{i}\left(x,y\right)}, \end{array}$$

where *β* is the gain adjustment coefficient and *α* is the nonlinear adjustment coefficient. MSRCR can get color fidelity and remove the color offset of the image.

After the luminance *V* component is enhanced, the saturation will also change accordingly, so the saturation component *S* should be corrected. In order to balance the saturation of the whole image and optimize the saturation of images with different illuminances, an adaptive stretch algorithm is adopted for saturation *S*. The saturation after stretching is obtained as follows:

(23) $$\begin{array}{c} \tilde{S}\left(x,y\right)=1+\left(\frac{M_{V}}{M+m+1}\right)\times S\left(x,y\right). \end{array}$$

*M*_*V*_ represents the average image saturation, *M* represents the maximum image saturation, and *m* represents the minimum image saturation. The drawing of formula (23) makes the images of different brightness enhanced. After the brightness of the image is enhanced, and the saturation is corrected in HSV space, the image can be enhanced by converting the image from HSV space to RGB space.

## 4. Experimental Verification and Result Analysis

In order to illustrate the feasibility and effectiveness of the algorithm, several haze images of different scenes are selected for enhancement processing, which will be verified and evaluated from subjective evaluation and quantitative analysis. The experimental environment includes Windows 10 operating system, 8G memory, 3.6 GHZ CPU, and MATLAB 2018. The image data used in this paper are all from the public data set and the data collected in the laboratory.

The subjective aspect is mainly based on human vision as the evaluation standard. In order to illustrate the applicability of the algorithm, different scene images with different haze concentrations in the research group image data set under natural conditions are selected for comparison of different algorithms. According to Figures 2–5, it can be seen that the defogging algorithm based on dark channel prior (DCP) has a certain degree of defogging after dark channel defogging, but the overall color is dark and has a certain distortion. The image enhanced by SSR, MSR, and MSRCR algorithms is prone to halo, edge blur and other phenomena on the edge of the image. With the deepening of the fog concentration, the defogging effect is getting worse and worse, the image quality is not clear, and the edge and other details of the sign are not obvious. Limited adaptive histogram equalization (CLAHE) can improve the contrast. Compared with DCP, CLAHE uses contrast limited processing in each neighborhood. CLAHE algorithm mainly enhances the local contrast to enhance the image details. The key of CLAHE algorithm is to restrict the contrast by clipping the histogram before calculating the conversion function: first, the original image is divided into several small blocks, then the histogram of each small block is calculated, and finally the histogram is redistributed by restricting the contrast of each small block. Although it improves the overall brightness, it enlarges the noise. The improved method of image enhancement has some improvement in color and edge. The new algorithm can effectively defog the high brightness areas such as the sky, and the contrast brightness of the whole image has been improved very well. The color of the image after defogging is more real, the details and certain scene depth are preserved, and the images are more natural.  Figure 6 is the gray histogram after image enhancement of this paper and Figure 7 is the comparison of running time of different algorithms.

Objective verification objective evaluation uses peak signal to noise ratio (PSNR), structural similarity index measurement (SSIM), and information entropy (IE) as the evaluation criteria between image enhancement algorithms.

The peak signal-to-noise ratio (PSNR) is an objective criterion used to evaluate the fidelity of an image. It is defined by the mean square error (MSE). If the PSNR is larger, the distortion of the image is smaller. The calculation process of peak signal-to-noise ratio is as follows: where *L* is the maximum gray value of the image.

(24) $$\begin{array}{c} \text{PSNR}=10\;\log_{10}\left(\frac{L^{2}}{\text{MSE}}\right). \end{array}$$

The structure similarity is a measure of the similarity between the defogging image and the original image, and the value range is [0, 1]. The larger the value is, the more complete the structure information of the original image is preserved, and the stronger the restoration ability of the defogging algorithm is. The calculation process of structural similarity is shown in formula (25), where *l*, *c* and *s* are the contrast functions of brightness, contrast and structure, and *α*, *β* and *γ* are the weights of the three functions, which are all positive numbers:

(25) $$\begin{array}{c} \text{SSIM}=l^{\alpha }c^{\beta }s^{\gamma }. \end{array}$$

Information entropy reflects the amount of information an image has. If the information entropy is larger, it means that the image has more information. The calculation process of information entropy is as follows: *M* is the total number of gray levels of the image, *P*_*i*_ is the probability of the pixel of the *i*-th gray level in the total pixel:

(26) $$\begin{array}{c} \text{IE}=-\sum_{i=0}^{M-1}P_{i}\;\log\;P_{i}. \end{array}$$

It can be seen from Table 1 and Figure 8 that the data through objective verification show that the improved algorithm is better than DCP, SSR, MSR, MSRCR, and CLAHE algorithm in PSNR, SSIM, and IE evaluation indexes in the case of haze, low illumination, and other interference factors. The image enhanced by the new algorithm has obvious improvement in brightness, contrast enhancement, noise removal, and anti-distortion. The experimental results show that the new algorithm can improve the image darkening, avoid image distortion, and has a good effect on preserving image edge information. It has good adaptability and stability, and is more suitable for fog image enhancement. The algorithm in this paper has good processing results in the haze world of low-quality road traffic images, the edge details of the enhanced results are more prominent, the reconstructed image has no color distortion and deviation, the image clarity and contrast have also been improved, the image noise has been weakened, and the prospective area has also been restored clearly, although the complete information of the image in sunny weather cannot be completely restored, but it can help restore image information and overall contour.

## 5. Conclusion

We breathe all the time. A person has to breathe more than 20,000 times a day and exchange at least 10,000 liters of gas with the environment every day. Haze weather will directly affect people's quality of life and health. In haze weather, there are a large number of particles, dust, pollutants, viruses, heavy metals, and other harmful substances floating in the air. When the human body inhales the haze through breathing, the toxic and harmful substances will invade the human respiratory tract and lungs. It will cause respiratory disease, cardiovascular disease, heart disease, and other diseases. Aiming at the problem that haze affects the image quality, an improved haze image enhancement method based on dark channel priority was proposed.

The new algorithm solved the problem that the dark channel prior method leads to the image color darkening, refines the transmittance, and optimizes the atmospheric light value. After restoration, the image was converted from RGB space to HSV space for secondary enhancement. In the process of enhancement, the *V* component was enhanced by MSRCR algorithm, and the saturation *S* was improved by adaptive stretching algorithm. Finally, the image was restored to RGB space, the haze image was defogged and enhanced. Objective image quality evaluation method is used to carry out quantitative evaluation. Information entropy, image gradient, and image variance are used as three indexes of image quality to evaluate the optimization effect of the algorithm. In the complex environment, the new method can significantly improve the brightness and contrast of the image, effectively remove the noise, suppress the image halo phenomenon, better enhance the color and clarity of the image, and improve the imaging effect. However, due to the low real-time performance of the algorithm in this paper, it cannot be applied to the system with high real-time requirements. Therefore, it is planned to further improve the real-time performance of the algorithm and expand the application scope of the system. In the follow-up research process, it should also consider the impact of image depth on the enhancement algorithm, use different enhancement coefficients for local areas with different depths, and consider its enhancement mechanism from many aspects. Therefore, we should make more in-depth research and improve it in the future.

## Figures and Tables

**Figure 1:** Algorithm flow.

**Figure 2:** Algorithms comparison of mountain. (a) Original image, (b) DCP, (c) SSR, (d) MSR, (e) MSRCR, (f) CLAHE, (g) the paper, and (h) dark channel.

**Figure 3:** Algorithms comparison of buildings. (a) Original image, (b) DCP, (c) SSR, (d) MSR, (e) MSRCR, (f) CLAHE, (g) the paper, and (h) dark channel.

**Figure 4:** Algorithms comparison of woods. (a) Original image, (b) DCP, (c) SSR, (d) MSR, (e) MSRCR, (f) CLAHE, (g) the paper, and (h) dark channel.

**Figure 5:** Algorithms comparison of traffic. (a) Original image, (b) DCP, (c) SSR, (d) MSR, (e) MSRCR, (f) CLAHE, (g) the paper, and (h) dark channel.

**Figure 6:** Gray histogram after image enhancement. (a) Gray histogram of mountain image, (b) gray histogram of building image, (c) gray histogram of woods image, and (d) gray histogram of traffic image.

**Figure 7:** Comparison of running time of different algorithms.

**Figure 8:** Comparison of image quality evaluation indexes.

**Table 1:** Performance comparison of image enhancement algorithms.

Evaluation criteria	Algorithms	Mountain	Buildings	Woods	Traffic
PSNR	DCP	17.131	20.651	21.745	18.356
	SSR	18.952	21.542	23.462	20.532
	MSR	20.349	23.747	25.854	22.646
	MSRCR	22.642	28.484	27.245	24.894
	CLAHE	24.958	26.102	26.457	25.461
	The paper	27.593	30.452	31.532	28.127

SSIM	DCP	0.067	0.075	0.082	0.071
	SSR	0.091	0.135	0.177	0.186
	MSR	0.206	0.228	0.332	0.316
	MSRCR	0.478	0.582	0.596	0.517
	CLAHE	0.513	0.682	0.641	0.701
	The paper	0.709	0.831	0.847	0.734

IE	DCP	10.542	11.245	12.935	11.523
	SSR	12.854	13.087	14.515	13.723
	MSR	15.778	15.961	16.274	14.852
	MSRCR	16.345	16.095	19.025	17.037
	CLAHE	17.154	17.549	19.574	17.562
	The paper	18.675	19.534	21.452	18.048

## Data Availability

The datasets used and/or analyzed during the current study are available from the corresponding author on reasonable request.
